# TiM-Net: Transformer in M-Net for Retinal Vessel Segmentation

**DOI:** 10.1155/2022/9016401

**Published:** 2022-07-11

**Authors:** Hongbin Zhang, Xiang Zhong, Zhijie Li, Yanan Chen, Zhiliang Zhu, Jingqin Lv, Chuanxiu Li, Ying Zhou, Guangli Li

**Affiliations:** ^1^School of Software, East China Jiaotong University, Nanchang, China; ^2^School of International, East China Jiaotong University, Nanchang, China; ^3^School of Information Engineering, East China Jiaotong University, Nanchang, China; ^4^Medical School, Nanchang University, Nanchang, China

## Abstract

retinal image is a crucial window for the clinical observation of cardiovascular, cerebrovascular, or other correlated diseases. Retinal vessel segmentation is of great benefit to the clinical diagnosis. Recently, the convolutional neural network (CNN) has become a dominant method in the retinal vessel segmentation field, especially the U-shaped CNN models. However, the conventional encoder in CNN is vulnerable to noisy interference, and the long-rang relationship in fundus images has not been fully utilized. In this paper, we propose a novel model called Transformer in M-Net (TiM-Net) based on M-Net, diverse attention mechanisms, and weighted side output layers to efficaciously perform retinal vessel segmentation. First, to alleviate the effects of noise, a dual-attention mechanism based on channel and spatial is designed. Then the self-attention mechanism in Transformer is introduced into skip connection to re-encode features and model the long-range relationship explicitly. Finally, a weighted SideOut layer is proposed for better utilization of the features from each side layer. Extensive experiments are conducted on three public data sets to show the effectiveness and robustness of our TiM-Net compared with the state-of-the-art baselines. Both quantitative and qualitative results prove its clinical practicality. Moreover, variants of TiM-Net also achieve competitive performance, demonstrating its scalability and generalization ability. The code of our model is available at https://github.com/ZX-ECJTU/TiM-Net.

## 1. Introduction

Artificial intelligence (AI) models have promoted the interactions between humans and computers greatly [1–3]. This phenomenon is more evident in the computer-aided diagnosis field. Recently, owing to the unhealthy living habits and growing pressure of life, the probability of people suffering from cardiovascular or cerebrovascular or other diseases has generally increased. From the medical perspective, the human eye is the only organ of the body that can directly observe the blood vessels and nerves. The retinal circulation has the same anatomical and physiological characteristics as the brain and coronary circulation. Hence, the retina of the human eyes has become an important window to diagnose cardiovascular, cerebrovascular, or other correlated diseases more efficiently. Traditionally, ophthalmologists make clinical diagnoses manually, which needs sufficient diagnostic experience and time. So the traditional diagnostic method is time-consuming and low efficient, which extends the corresponding diagnostic cycle with much financial and mental pressure on the patients. With the rapid development of AI technologies, more and more doctors began to use computer-aided diagnosis (CAD) methods to alleviate this problem. The realization of the CAD-based retinal vessel segmentation method helps the ophthalmologists more accurately and efficiently observe retinal diseases [4] and also allows the patients to receive higher quality treatments. Since 2012, deep learning methods, such as convolutional neural network (CNN) [5] and recurrent neural network, have greatly promoted the development of the computer vision (CV) field. More and more CV tasks using specific CNN structures can obtain state-of-the-art performance. Recently, fully connected networks [6], U-Net [7], and U-Net++ [8] have become the dominant methods in medical image segmentation. The U-Net and U-Net++ models, usually use a symmetric encoder-decoder framework with skip connections to enhance the quality of detail retention. U-Net is simple, but it builds a firm foundation for the subsequent correlated research. Hence, many methods based on U-shaped networks were proposed to complete medical image segmentation, and they achieved great success in numerous tasks, such as retinal vessel segmentation [9–12], heart segmentation [13], and organ segmentation [10, 14].

Recently, deep learning models have played a very important role in retinal vessel segmentation [15, 16] owing to their high practicality. Fu et al. [17] added a multiscale input layer to U-Net as well as a side output layer. However, feature filtering was not implemented in the skip connections of the M-Net model, and each side output layer uses the same weight. Guo et al. [18] placed the spatial attention module behind the encoder to extract significant features. Only using spatial attention loses the key information across different feature channels. Fu et al. [19] used parallel channel and spatial attention to suppress the negative influence of noisy features. Zhang et al. [20] absorbed a gate attention mechanism into the skip connection for filtering noisy information. Wang et al. [21] designed a hard attention network (HA-Net) consisting of three decoders for retinal vessel segmentation. Li et al. [22] adopted the weight-sharing and skip-connection features to facilitate training. The pyramid U-Net [23] acquires aggregated features at higher, current, and lower levels in its encoder and decoder. Recently, owing to the great success of Transformer in the CV field, TransUNet [24] and TransFuse [25] have been proposed by combining Transformer and U-Net. Similarly, Chen proposed the patches convolution attention-based Transformer U-Net (PCAT-UNet) [26] model that inserts a modified Transformer module into U-Net. Although better performance can be observed, these Transformer-based models are complex and time-consuming, which will affect their practicalities to some degree.

Based on the above analysis, we found the following difficulties of previous work: (1) it is difficult to obtain the best performance on each evaluation metric; (2) it is difficult to combine the Transformer module and U-Net model owing to the high complexity; (3) feature maps are prone to noise interference; (4) it is difficult to effectively model the long-range relationships in the fundus images; and (5) the output layers only use one single layer, which did not exploit the utility of other layers.

This study focuses on the (3), (4), and (5) problems. We first design a novel dual-attention mechanism and then apply it to our model. The dual-attention mechanism can effectively alleviate the interference of noisy information. Second, we explicitly model the long-rang relationship in the fundus images by using a pure Transformer module. Both the proposed dual-attention mechanism and Transformer module are plug-and-play, making our model simple and easy to implement. Finally, we assign a suitable weight to each side output layer based on its real importance. We are striving to make full use of the complementarity of multiple output layers. Conceptually and empirically, the main contributions of this paper can be summarized as follows:

1. We propose a novel model called Transformer in M-Net (TiM-Net), which is simple but effective for retinal vessel segmentation. TiM-Net takes multiscale input, feature refinement strategies, and long-range relationship into account, which can strengthen the discriminative abilities of image features. TiM-Net achieves satisfactory segmentation results, which provides firm technical support for clinical human-computer interaction diagnosis.
2. Extensive experiments were conducted on three public benchmark data sets. The corresponding results demonstrate the superior segmentation performance of TiM-Net over other state-of-the-art methods. The code of our model is available at https://github.com/ZX-ECJTU/TiM-Net.
3. Owing to a relatively flexible structure, TiM-Net has several model variants. These model variants also obtain competitive segmentation performance, demonstrating the powerful scalability and generalization ability of TiM-Net.
4. We complete both coarse- and fine-grained ablation analysis to evaluate the real contribution of each module in TiM-Net, which provides a new idea for evaluating the segmentation model comprehensively.

The remainder of this paper is organized as follows: Section 2 presents related work and our research motivations. TiM-Net is described in Section 3. Experiments on three well-known retinal image data sets and the corresponding results are discussed in Section 4. Finally, Section 5 provides the conclusions and our future work.

## 2. Related Work

### 2.1. Medical Image Segmentation

In the traditional U-shaped segmentation models, the encoders usually employ two methods, including superimposed convolutional layers and continuous down-sampling, to generate a sufficiently large receptive field, thus improving the efficiency of global context modeling. However, these methods bring the following drawbacks: (1) The features extracted from the encoders contain many noises, which affect the final segmentation performance, and (2) their models using too many parameters are prone to overfitting when the corresponding medical image data set is relatively small. To address these problems, some researchers used additional expansion paths to better extract both coarse- and fine-grained features for segmentation. For example, Zhang et al. [27] introduced three different dense connections in multiscale densely connected U-Net to combine the features from different scales. Feature fusion was carried out, in turn, to strengthen the discriminative ability of the features and reduce the risk of overfitting. Chen et al. [28] proposed a bridging method to connect two U-Net structures, which can make full use of the features extracted from the two networks. Devi et al. [29] embedded a multiscale dilated convolution module in the decoders to fuse multiscale features for automatic instrument segmentation. In summary, the U-shaped model is the mainstream model in the medical image segmentation field.

### 2.2. Attention Mechanism

Owing to noisy interference, some important edge information is ignored by the segmentation model. And the corresponding performance is unsatisfactory, especially for retinal vessel segmentation. To address this problem, more and more researchers added the well-known attention mechanism [30] to U-Net. They want to capture the most correlated features for effective medical image segmentation. Li et al. [31] inserted a gate attention mechanism to the skip connection of U-Net. It focuses on the position of the encoded features in the target area. Unlike the single attention mechanism, the dual-attention mechanism [19, 32, 33] has been proposed to choose the most significant channel features and suppress irrelevant spatial features. Wang et al. [34] used the dual-attention mechanism combined with residual connection in the encoder and decoder structures. Experiments demonstrate that the combination of channel and spatial attention outperforms a single attention mechanism. Fu et al. [17] used parallel channel and spatial attention to suppress the negative influence of noisy features. Amer et al. [35] proposed a multiscale spatial attention module in which the spatial attention graph is derived from a hybrid hierarchical dilated convolution module. This module can capture multiscale context information for lung image segmentation. Summarily, extensive experiments have validated the effectiveness of the attention mechanism in medical image segmentation.

The Transformer uses another kind of attention mechanism. It has pioneered new technologies in the fields of machine translation [36] and natural language processing [37]. Evident performance improvement can be observed on numerous tasks. Notably, lots of studies have demonstrated that Transformer is also suitable for CV tasks. Dosovitskiy et al. [38] implemented the well-known vision Transformer (ViT), directly applying the Transformer and the global self-attention mechanism to classify full-size images. Ye et al. [39] proposed a cross-modal self-attention mechanism that incorporates image and text features for query, key, and value. Yang et al. [40] proposed a cross-scale feature integration module that learns more powerful feature representations by stacking multiple texture Transformers. Liu et al. [41] proposed a hierarchical Transformer that limited self-attention computing to nonoverlapping local windows while allowing the cross-window connection.

Recently, some researchers began to introduce Transformer into the medical image segmentation field and obtained satisfactory performance. The Transformer converts each image into a one-dimensional sequence and focuses on modeling the global context. Chen et al. [24] proposed the TransUNet model that replaces the encoder of the U-Net model with a Transformer structure. Zhang et al. [25] designed the TransFuse method that fuses Transformer with CNN. The two models obtained evident performance improvement in medical image segmentation. However, the two models are very complex.

### 2.3. Retinal Image Segmentation

This study focuses on retinal vessel segmentation. For this task, Fu et al. [17] added a multiscale input layer into U-Net as well as a side output layer, which solves the segmentation problem of the optic disc and optic cup. Wang et al. [42] proposed a double-coded U-Net model and placed the channel attention on the skip connection to choose effective features. Ma et al. [43] proposed a multitask CNN with a spatial activation mechanism, which can simultaneously segment retinal blood vessels, arteries, and veins. Guo et al. [18] put a spatial attention module at the bottom-most layer of an encoder for adaptive feature refinement. This attention module can suppress the uncorrelated features to some degree. Zhang et al. [20] absorbed a gate attention mechanism to the skip connection. Wang et al. [21] designed the HA-Net model consisting of three decoders. The first decoder can dynamically analyze the “hard” and “easy” regions of the image, while the other two decoders are responsible for distinguishing the “hard” and “easy” regions of the retinal blood vessels. Tong et al. [44] proposed a side attention network that integrated side-attention and dense atrous convolutional blocks, preserving more features of the encoder and contextual information of the fundus image, respectively. Li et al. [22] adopted the weight-sharing and skip-connection features to facilitate training. Jiang et al. [45] used both multiscale dilated convolution and skip connection to reduce the loss of feature information. Zhai et al. [46] used multiple pyramid pooling modules to combine more contextual information in the decoding process. Zhang et al. [47] proposed a structure-texture demixing network for separating structure and texture components, which can better handle structure and texture in different ways. Cao [48] proposed a pure Transformer network to classify and segment images with great success. Chen et al. [26] proposed the PCAT-UNet model that absorbs a modified Transformer module into U-Net. However, due to the lack of the ability to capture the long-range relationship, noisy features are obtained after multiple convolutions, which affects the final performance.

### 2.4. Motivations

Reviewing the work of [17, 18, 24–26], we found the following problems: (1) most studies use complex structures, which may lower their practicalities; (2) traditional encoders cannot model long-range relationships and are prone to noisy interference; and (3) the side output layer only uses a single-layer output, which cannot make full use of the complementarity of different layers. The complementarity helps recover the feature maps well.

Hence, our motivations are threefold. First, to lower complexity, we consider a plug-and-play approach that only adds a Transformer to skip connection. Second, unlike the M-Net model, we incorporate diverse attention mechanisms, including the self-attention of Transformer and dual-attention mechanism, into two different positions of our model. On the one hand, we absorb the Transformer module into the skip connection to re-encode the image features extracted from the encoder. This can refine the encoded features to a certain degree. More importantly, this helps explicitly model the long-range relationship in the fundus images. On the other hand, we propose the dual-attention mechanism including spatial attention and channel attention to reduce the negative effect of the noisy features. Lastly, we make full use of each side layer through a suitable weight assignment strategy. All these modifications are easy to implement and cannot increase the complexity of the segmentation model, which also contributes to promoting the practicality of TiM-Net.

## 3. Method

Problem definition: Our goal is to predict the corresponding label map with the size of *H* × *W* × *C* of an arbitrary retinal image. *H* is the height of the image. *W* is the width of the image. *C* is the corresponding channel number. Our model is illustrated in Figure 1.

First, TiM-Net uses multiscale images as its input. This can leverage the multiscale information for retinal vessel segmentation. Second, TiM-Net incorporates the Transformer module into its skip connection. The built-in self-attention mechanism of the Transformer models the long-range relationship in the fundus images and makes effective feature refinement. This builds a firm foundation for the subsequent upsampling. Third, the dual-attention module including spatial and channel attention is placed behind the last encoder layer to prevent gradient degradation and make another kind of feature refinement. Finally, we make full use of each side layer to complete the final segmentation. We introduce each component as follows.

### 3.1. Transformer in Skip Connection

The traditional attention mechanism uses different input sources and output targets, which has a certain negative influence on feature decoding. Moreover, it cannot model the long-range relationship in the fundus images. As we know, the Transformer employs the self-attention mechanism, which has the same target and source. More importantly, this self-attention mechanism can better model the long-range relationship across a whole image. Hence, we absorb the Transformer module into the skip connection at a suitable position. The corresponding structure of the Transformer is shown in Figure 2.

In Figure 1, the second layer features extracted from the encoder are input into the Transformer to implement self-attention computing. The corresponding results are transferred into the decoder. Hence, we absorb the Transformer module into the skip connection. The Transformer divides the input feature maps (256 × 256) into 16 patches, namely *p*^*i*^, averagely, and each patch size is *P* × *P*. Then these patches are serialized and passed into the embedding layer to obtain the original embedding sequence. They are linearly projected to a *D*-dimensional embedding space in turn.

To learn specific spatial information about these patches, position embeddings are first added to the patches to preserve position information. Then the built-in self-attention mechanism in the Transformer module calculates the correlation between each patch pair. Finally, the spatial correlation of given patches is obtained through a multilayer perceptron (MLP) layer. Position embeddings are used as follows:

(1) $$\begin{array}{c} z_{0}=\left\{p^{1}X;p^{2}X;\ldots ;p^{16}X\right\}+X_{\text{pos}}, \end{array}$$

where *X* ∈ *ℜ*^(*P* × *P* × *C*)×*D*^ denotes the matrix that implements the corresponding linear projection as illustrated in Figure 2(a). *p*^*i*^*X*(i ∈ {1,&,16}) denotes a linear projection result of *p*^*i*^. **X**_pos_ represents the corresponding position embedding of the given patches, so the position information of each patch is reserved by marking the original position serial number of *p*^*i*^. This contributes to learning global long-range relationships in the fundus images. According to equation (1), the Transformer makes a linear projection of *p*^*i*^ and forms a *D*-dimensional *z*_0_ together with position embedding. This can also be regarded as a kind of preprocessing step for the subsequent self-attention computing. It builds a foundation for capturing long-range relationships in the fundus images.

The projections are input into the encoder layer of the Transformer, which contains *n* layers of multihead self-attention (MSA) and MLP. The detailed structure of the encoder layer is illustrated in Figure 2(b). Therefore, the output of the *n*-th layer can be calculated as follows:

(2) $$\begin{array}{c} z_{n}^{\prime }=\text{MSA}\left(LN\left(z_{n-1}\right)\right)+z_{n-1}, \end{array}$$

(3) $$\begin{array}{c} z_{n}=\text{MLP}\left(LN\left(z_{n}^{\prime }\right)\right)+z_{n}^{\prime }, \end{array}$$

where *z*_*n*_ denotes the encoded image sequence and *LN* denotes the normalization layer. Finally, the output feature is reshaped to its original size. Owing to MSA and MLP, the Transformer can model the long-range relationship well and further refine the extracted features. Summarily, equation (3) makes the MLP projection of the results of self-attention computing and generates the refined image features for the subsequent upsampling operations.

### 3.2. Dual-Attention Mechanism in Encoder

Deep learning features acquired through multiple convolutions inevitably mix numerous noisy features. Meanwhile, gradient degradation usually occurs when the segmentation model is too deep. Hence, we need to make feature refinement and strengthen the feature propagation procedure. To resolve the two problems, we place the dual-attention mechanism behind the encoder layer to suppress the noises and promote model optimization. The proposed dual-attention module is shown in Figure 3.

As shown in Figure 3, channel attention focuses on “what” is meaningful in the input image, whereas spatial attention focuses on “where” is the most informative region. The two attentions complement each other. Experiments in [33] have demonstrated that sequential channel attention and spatial attention are effective. Unlike [33], we add the residual links after the convolution layer rather than before. This strategy has two evident advantages: First, it ensures the same number of channels. Second, it makes the whole procedure more efficient. Hence, each kind of attention mechanism captures the most important features from its perspective. And they complement each other to make more effective feature refinement.

Here, we give the formal description of the dual-attention mechanism. It first obtains the feature map *F* ∈ *ℜ*^*C*×*H*×*W*^ through a 1 × 1 convolution and then gets the channel attention feature map *F*_*c*_ ∈ *ℜ*^*C*×1×1^. After *F*_*c*_ multiplying *F*, the spatial attention feature map *F*_*s*_ ∈ *ℜ*^1×*H*×*W*^ is acquired. Finally, we get the last feature map *F*′ ∈ *ℜ*^*C*×*H*×*W*^. It represents the final output of the dual-attention mechanism. The detailed equation of the dual-attention mechanism is shown as follows:

(4) $$\begin{array}{c} F{}^{\prime }=F+F\times F_{c}\left(F\right)\times F_{s}\left(F\times F_{c}\left(F\right)\right). \end{array}$$

Equation (4) represents the output of the dual-attention mechanism, which can suppress the noisy information in the encoded features. The following two subsections present channel attention and spatial attention, respectively.

#### 3.2.1. Channel Attention

In this subsection, we mine the relationship between different channels to obtain channel attention. We intend to find the channels that contain more valuable information for retinal vessel segmentation. Hence, the channel attention mechanism can retain the key information to the most extent. The channel attention employs the global average pooling and global max-pooling layers to squeeze the feature maps in the spatial dimension. The global average pooling layer captures the overall information of image features, whereas the global max-pooling layer obtains the difference information of these features.  Figure 4 illustrates the core idea of channel attention.

As shown in Figure 4, we implement global max-pooling (Maxpool) and global average pooling (Avgpool) on the input feature map *F* ∈ *ℜ*^*C*×*H*×*W*^, respectively. Two feature maps, namely *F*_avg_^*c*^ and *F*_max_^*c*^, are obtained. The two feature maps are input into a two-layer MLP. The neuron number of the first layer in the MLP is *C*/*r*, where *r* is the decay rate. The neuron number of the second layer in the MLP is *C*. The MLP model uses RELU as its activation function. Finally, the element-wise summation is implemented based on the two outputs of the MLP model, namely *F*_1_ and *F*_2_. Sigmoid is chosen to generate the final channel attention feature maps *F*_*c*_. Hence, the whole procedure of the channel attention can be formulated as follows:

(5) $$\begin{array}{c} F_{c}=\sigma \left(\text{MLP}\left(\text{Avgpool}\left(F\right)\right)+\text{MLP}\left(\text{Maxpool}\left(F\right)\right)\right)=\sigma \left(W_{1}\left(W_{0}\left(F_{\text{avg}}^{c}\right)\right)+W_{1}\left(W_{0}\left(F_{\text{max}}^{c}\right)\right)\right), \end{array}$$

where *F*_avg_^*c*^ and *F*_max_^*c*^ represent the output of the two pooling layers, respectively. *σ* is the Sigmoid activation function. *W*_0_ ∈ *ℜ*^*C*/*r*×*C*^ and *W*_1_ ∈ *ℜ*^*C*×*C*/*r*^ represent the corresponding weights of the MLP model, which are shared for each output of the pooling layer. *F*_*c*_ represents the acquired channel attention feature map, which mainly depicts the valuable information in different feature channels.

#### 3.2.2. Spatial Attention

As described above, the channel attention module focuses on capturing the key information among different channels. As illustrated in Figure 5, unlike the channel attention module, spatial attention emphasizes the key segmentation information hidden in the spatial dimension more.

We implement global max-pooling and global average pooling on the input feature maps *F*′ generated by the channel attention module. Two feature maps, namely *F*_avg_^*s*^ and *F*_max_^*s*^, are obtained in turn. They pay more attention to the local key regions in the fundus images. We concatenate the two feature maps and implement a 7 × 7 convolutional operation named *f*^7×7^, where the padding is 3. The sigmoid function is chosen to generate the final spatial attention feature maps. Hence, the whole procedure of the spatial attention can be formulated as follows:

(6) $$\begin{array}{c} F_{s}=\sigma \left(f^{7\times 7}\left(\begin{array}{c} \left[\text{Avgpool}\left(F{}^{\prime }\right)\right]\\ \left[\text{Maxpool}\left(F{}^{\prime }\right)\right] \end{array}\right)\right)\\ =\sigma \left(f^{7\times 7}\left(\left[F_{avg}^{s};F_{\max}^{s}\right]\right)\right), \end{array}$$

where *F*_avg_^*s*^ and *F*_max_^*s*^ represent the output of the two pooling layers. *σ* is the Sigmoid activation function. *F*_*s*_ represents the feature map generated by spatial attention, which mainly highlights the key spatial information hidden in feature maps for blood vessel segmentation.

### 3.3. TiM-Net

TiM-Net derives from M-Net [17]. Hence, it consists of the M-Net architecture, a new encoder combined with the dual-attention mechanism (left side), the Transformer-based skip connection that transfers the refined features to the decoder, and a new decoder combined with a group of weighted side output layers. Please refer to Figure 1 to get the detailed structure of TiM-Net.

In our encoder, we first use max-pooling to downsample the retinal vessel images and construct multiscale inputs for encoding. This strategy has two advantages: (1) multiscale images offer more sufficient information to depict vessel details and (2) it avoids the large growth of parameters and makes TiM-Net prone to reproduce. Then we place the dual-attention mechanism behind the encoder to suppress noisy information. The dual-attention mechanism is made up of the channel and spatial attention modules. They complement each other and adaptively reassign suitable weights to the corresponding encoded features.

Unlike TransUNet and TransFuse, we need not modify the whole encoder. We only absorb the Transformer module to the skip connection. We intend to re-encode feature maps and capture the long-range relationship in the fundus images. Multiple image blocks are extracted and input into the modified skip connection to complete feature re-encoding. We make full use of the MSA mechanism of the Transformer module to further re-encode these feature maps. Owing to the self-attention characteristic, the long-range relationship among diverse feature patches is mined out. It is a significant complementarity to the local region-based convolutional information.

In our decoder, we use four side layers to construct different outputs. Each side layer depicts the segmented results from its perspective. They complement each other. To directly utilize the predicted maps of each side layer, we combine the loss *L*_*i*_ of each side layer and create the final loss *L* as shown in (7). Each side layer is weighted by *α*_*i*_(*i*=1,2,3,4), respectively. We tune these weights carefully (please refer to Table 7). This can backpropagate the loss of each side layer and the final loss to the earlier layers of the decoder, which helps alleviate the gradient degradation problem. Moreover, we take full advantage of each side layer to obtain better segmentation results. The output loss function *L* is defined as follows:

(7) $$\begin{array}{c} L\left(V,v\right)=\sum_{i}^{M}\alpha_{i}L_{i}\left(V,v^{\left(i\right)}\right), \end{array}$$

where *M* is the output number. *L*_*i*_ is the loss of the *i*-th side output layer. Accordingly, *v*^(*i*)^ denotes the weight of the *i*-th side output layer. *V* represents the parameters of all the standard convolutional layers.

## 4. Experiments

### 4.1. Data Sets and Evaluation Metrics

In this section, extensive experiments are conducted to verify the effectiveness and generalization ability of TiM-Net on three public data sets, including STARE [49], CHASEDB1 [50], and DRIVE [51].

1. STARE: It is a color image data set used for retinal vessel segmentation, which includes 20 retinal images. Ten images of this data set are diseased, whereas another 10 images have no disease. The image resolution is 605 × 700. We randomly select 14 images for training and other 6 images for evaluation. From the perspective of disease distribution, STARE is a balanced data set, which indicates that it is relatively easier to train the corresponding segmentation model.
2. CHASEDB1: It is a 999 × 960 image data set containing 28 retinal images of the central nervous vascular reflex. No image contains disease. We use 20 images for training and other 8 images for evaluation. Unlike the other two data sets, the corresponding image size of CHASEDB1 is larger, which indicates that we need to capture sufficient long-range relationships for better segmentation.
3. DRIVE: It includes 40 images. Seven images in this data set are early diabetic retinopathy, whereas another 33 samples are the fundus images without diabetic retinopathy. The resolution of each image is 565 × 584. We divide the training set and test set into 1:1. Unlike the above two data sets, it is an imbalanced data set, which means a relatively more challenging segmentation task. But it is closer to clinical conditions.

According to the above presentation, all the data sets cover diverse diseases, data distributions, and image sizes. This setting has two advantages: (1) this can firmly validate the effectiveness and robustness of our segmentation model and (2) this can objectively mimic the real clinical diagnosis procedure to some degree.

Similar to most methods of retinal image segmentation, we use the accuracy (Acc), sensitivity (Se), specificity (Sp), and area under ROC (AUC) metrics to evaluate each segmentation model. Acc is used to evaluate the overall segmentation performance of the model. Larger Acc means that both objects (vessel or background) can be segmented accurately. It is shown as follows:

(8) $$\begin{array}{c} \text{Acc}=\frac{\text{TP}+\text{TN}}{\text{TP}+\text{TN}+\text{FP}+\text{FN}}. \end{array}$$

Se is another important metric of retinal vessel segmentation. It is the ratio of correct positive predictions to the total number of positive predictions in the predicted results. This metric mainly evaluates the ability to recognize retinal vessels (positive) in retinal images. The better the Se value, the lower the false negative rate (FNR). The Se metric is shown as follows:

(9) $$\begin{array}{c} \text{Se}=\frac{\text{TP}}{\text{TP}+\text{FN}}. \end{array}$$

Sp is another mainstream metric of retinal vessel segmentation. It is the ratio of correct negative predictions to the total number of negative predictions. It mainly evaluates the ability to recognize background (negative) in retinal images. The better the Sp value, the lower the false positive rate (FPR). Hence, the Sp metric is shown as follows:

(10) $$\begin{array}{c} \text{Sp}=\frac{\text{TN}}{\text{TN}+\text{FP}}. \end{array}$$

Here, TP, TN, FP, and FN denote the number of true positives, true negatives, false positives, and false negatives, respectively.

In addition, we introduce the AUC metric to evaluate the segmentation performance of each model. It is an important overall metric. A larger AUC indicates satisfactory performance, which indicates that the corresponding ROC curve is very close to the (0, 1) point and far from the 45° diagonal of the coordinate axis.

We used the PyTorch backend to implement all networks. We conducted all the experiments on our computer server with four NVIDIA GeForce GTX 2080Ti GPUs. We only need to resize each original image to 512 × 512. The learning rate is 0.0015, and the batch size is 2. We compare the TiM-Net model with numerous state-of-the-art methods. We use Acc, Se, Sp, and AUC metrics to evaluate each model more comprehensively.

### 4.2. Experimental Results

#### 4.2.1. Quantitative Results on STARE

In this section, we make detailed performance comparisons. We first show the corresponding comparisons on STARE in Table 1. We use two variants, namely TiM-Net-1 and TiM-Net-2, in this experiment. TiM-Net-1 means that only Side7 is chosen as the final prediction. TiM-Net-2 represents that SideOut is the final prediction layer.

As shown in Table 1, TiM-Net-2 obtains the best Se and Acc on STARE. Highly competitive Sp and AUC can be observed too. First, the best Se, especially for TiM-Net-1, means that TiM-Net can more accurately identify retinal vessels (positive), which represents the best FNR among all the models. More blood vessels can be offered for clinical diagnosis and produce the effect. As described above, the MSA mechanism of the Transformer module focuses on capturing the foreground global vessel details. And the dual-attention mechanism can suppress noisy interference well. These two factors positively boost the FNR value. Second, highly competitive Sp indicates that TiM-Net has a very competitive FPR. Noisy information is suppressed to a certain degree, which can improve the practicality of TiM-Net and effectively assist in doctors' clinical diagnoses. Although reference [54] gets the best AUC, TiM-Net-2 outperforms it on any other metric. Compared with [17, 54, 55], relatively higher overall performance is obtained using TiM-Net-2. Certainly, the AUC value of our model needs further improvement. Summarily, each model variant is effective for retinal vessel segmentation on STARE, demonstrating its better scalability and generalization ability.

#### 4.2.2. Quantitative Results on CHASEDB1

We show the corresponding comparisons on the CHASEDB1 data set in Table 2. We also use the two variants introduced above.

As shown in Table 2, TiM-Net-2 gets the best Acc and Sp, competitive Se, and AUC. The best Acc means that both objects (vessels or background) can be segmented accurately. More vessel details are offered for clinical diagnosis. The best Sp indicates that TiM-Net has the best FPR. The background (negative) of the CHASEDB1 images is better segmented. And doctors can get more evident pathological observations. Although reference [21] obtains the best AUC, TiM-Net-2 outperforms it on both Acc and Sp metrics. Compared with [55], TiM-Net-2 achieves superior performance on the other three metrics except for Se. Our model is relatively competitive for retinal vessel segmentation on CHASEDB1. However, the Se metric of TiM-Net needs further improvement. Some vessels are wrong and recognized as the background. This is mostly due to the visual similarity between the background and vessels. To solve this issue, we may do some data preprocessing steps. Currently, we have achieved satisfactory results without such preprocessing steps. Moreover, we will further focus on feature learning using some state-of-the-art methods, such as MAE [57] and ViT [38]. Summarily, our model is effective for retinal vessel segmentation on the challenging CHASEDB1 data set.

#### 4.2.3. Quantitative Results on DRIVE

We show the corresponding comparisons on the DRIVE data set in Table 3. We use the two variants introduced above.

As shown in Table 3, TiM-Net-2 obtains the best Acc and the other three competitive values on DRIVE. More vessel details are offered for clinical diagnosis. And the background (negative) of the DRIVE image is better segmented by TiM-Net. Although reference [7] obtains the best Sp, TiM-Net-2 outperforms it on all other metrics. Similarly, although reference [21] gets the best Se and AUC, TiM-Net-2 beats it on other metrics. Our model is relatively competitive on the imbalance data set. It can generate sufficient effective information for clinical diagnosis. Certainly, some vessels are segmented as the background, which leads to low Se (please refer to TiM-Net-1; the best Se will be obtained if we choose the Side7 layer, which demonstrates the scalability of TiM-Net to some degree).

Summarily, the above results demonstrate the effectiveness, robustness, and scalability of TiM-Net. It achieves the best overall performance on three public data sets. Unlike other models, such as [7, 9, 21, 41, 55] and so on, which need preprocessing steps, our model achieves satisfactory results without such steps. Owing to very competitive performance, TiM-Net offers sufficient information for the actual diagnosis.

#### 4.2.4. Qualitative Results

In this section, we use one representative retinal vessel image from each data set as an example to more intuitively show the corresponding qualitative segmentation performance. Similar results can be observed when we use other images. The morphological characteristics of the segmented retina can be used to assist doctors in the diagnosis of diabetic retinopathy, glaucoma, and age-related macular degeneration. The qualitative results are shown in Figures 6 and 7. We compare our model with M-Net and U-Net.

As shown in Figure 6, we choose some representative local regions to zoom in. The hard regions are mainly composed of thinner blood vessel boundaries, whereas the easy regions are made up of thicker blood vessel boundaries. Owing to MSA, sufficient long-range relationship in the fundus images is captured accurately to decode the key blood vessel boundaries, especially for the CHASEDB1 data set. Compared with U-Net, TiM-Net owns superior performance for both easy and hard regions on STARE. Similar results can be observed on DRIVE and CHASEDB1. Compared with M-Net, our model has obvious advantages for thinner blood vessels on DRIVE. More vessel details are precisely segmented by TiM-Net, which can assist doctors in observing lesion areas and making accurate diagnosis decisions. Certainly, the corresponding performance on small blood vessels needs further improvement. Summarily, TiM-Net obtains the best overall qualitative segmentation performance, which firmly supports the clinical diagnosis.

As shown in Figure 7, to further explore the clinical practicality of TiM-Net, we compare the segmentation results of disease and nondisease cases on DRIVE. We choose some representative local regions to zoom in. The disease cases usually have more noise, and the blood vessels in the hard regions are more blurred than those in the nondisease images. Hence, accurate blood vessel segmentation has significant clinical value. Moreover, this has a certain influence on the segmentation result. First, by observing the segmentation results of the disease images, we found that our model had an advantage in obtaining more vascular details, which can assist doctors in observing the lesions and making correct diagnostic results. We conclude that this is mostly due to the combination of the MSA and dual-attention mechanisms. Second, by observing the segmentation results of the nondisease images, we found that although TiM-Net owns better segmentation results than other models, there is no evident advantage because each nondisease image has clearer vessel details. Summarily, our model can better obtain the implicit relationship between feature channels and long-range relationship in the fundus images, to segment disease images accurately, which has significant clinical value.

### 4.3. Other Optimizations

We use a group of side output layers, including Side5, Side6, Side7, Side8, and SideOut, to complete the final segmentation prediction. Each side layer can be employed to make segmentation independently. Then, we complete feature fusion using all the layers. So the SideOut layer represents the weighted sum of each side layer. The weight *α*_*i*_ (*i* = 1, 2, 3, 4) of each side layer is set equally (0.25). And we obtain the corresponding experimental results shown in Table 4. We use Acc, Se, Sp, and AUC metrics to evaluate the model.

As shown in Table 4, on each data set, Side8 outperforms Side5, Side6, and Side7 on the Sp and Acc metrics. The phenomena are more evident on CHASEDB1. This means that more significant information is decoded at the last side layer, which helps improve the final performance. However, the AUC of Side8 is unsatisfactory, especially for CHASEDB1. Side8 is a relatively better choice if we only need a lower FPR. Second, Side7 outperforms Side5 and Side6 on the Acc, Se, and Sp metrics. The phenomena are more evident on CHASEDB1. Much valuable information is still retained in the Side7 layer. It is a firm foundation for the final prediction. Similar to Side8, Side7 is another good choice if we focus on a specific metric, such as Se or Acc. Moreover, SideOut gets the best AUC and competitive Acc and Sp. All these results demonstrate that different side layers complement each other and they create a kind of joint force to boost the final performance. Overall, the SideOut layer obtains a more balanced performance among all the side layers.

According to the results of Table 4, we get the following to ascend rank order of all the side layers: “Side5 < Side6 = Side7 < Side8.” Hence, we must set different weights for different side layers to further improve segmentation performance. We tune *α*_*i*_ (*i* = 1, 2, 3, 4) to 0.10, 0.25, 0.25, and 0.40, respectively. We use Acc, Se, Sp, and AUC metrics to evaluate each model. All the results are shown in Table 5. Moreover, to observe the performance improvement of each layer, we average the corresponding performance improvement of each metric on all the data sets compared to Table 4 and draw Figure 8.

As presented in Table 5, on each data set, Side8 outperforms Side5, Side6, and Side7 on the Sp and Acc metrics. The phenomena are more evident in the STARE and DRIVE data sets. This means that sufficient important information is decoded accurately at the last side layer. Certainly, the AUC of Side8 is unsatisfactory. Side8 is a relatively optimal choice if we need the best overall performance or a lower FPR. Second, Side7 outperforms Side5 and Side6 on most metrics. The phenomena are more evident in DRIVE and STARE. Much valuable information is retained in Side7. It is another firm foundation for weighted prediction. Moreover, the SideOut layer gets the best AUC and Acc. The best overall performance is obtained by assigning a suitable weight to each side layer. Different side layers complement each other and create a kind of joint force to boost the final performance.

It is worth noting that compared with Table 4, more improvements of SideOut are found in Table 5. Four metrics get performance improvements on STARE and CHASEDB1, whereas three metrics get more evident improvements on DRIVE. These results validate that we must use those significant features to complete the final segmentation. Meanwhile, different side layers complement each other and contribute to boosting the final performance from their views. As another suitable choice, we can choose Side7 if we focus on improving a specific metric, such as Se or Acc (please refer to the results of TiM-Net-1 in Tables 1–3). This demonstrates the effectiveness of TiM-Net from another perspective.

As shown in Figure 8, from the perspective of Se, the best performance improvement was achieved when Side8 was chosen. From the perspective of Sp and Acc, Side5 achieves the best improvement, which indicates that it has better segmentation accuracy and a lower FPR. The model variant using Side5 segments blood vessels more correctly. However, this model requires a great sacrifice of vascular segmentation performance. In terms of AUC, Side7 achieves the best performance improvement, which implies that Side7 can distinguish negative and positive objects well. Overall, SideOut achieves relatively better and more balanced performance improvement, and its performance is more robust and satisfactory, which could firmly support clinical diagnosis.

Summarily, on the one hand, the SideOut layer obtains a more balanced segmentation performance. On the other hand, the best overall performance is obtained by setting a suitable weight for each side layer. Different side layers complement each other to boost the final performance. Therefore, the TiM-Net model employs the new weighted SideOut layer to make the final retinal vessel segmentation.

### 4.4. Ablation Analysis

In this section, we complete a group of detailed ablation analyses, including the application of the Transformer module (Subsection 4.4.1), and the real contribution of each module in TiM-Net (Subsection 4.4.2).

#### 4.4.1. Application of Transformer

To validate the effectiveness of the modified skip connection, we make the following experiments. We add the Transformer module into the second layer (TransL2), third layer (TransL3), and fourth layer (TransL4). We want to know where the best position is to apply the Transformer module and how many Transformer modules are needed for TiM-Net. We use Acc, Se, Sp, and AUC metrics to complete our experiments. All the results are shown in Table 6.

As shown in Table 6, for DRIVE and CHASEDB1, the largest performance improvement can be observed in TransL2. This means that effective feature learning or feature selection by the Transformer module is obtained at the top layer, which contains much more valuable discriminative information and long-range relationship in the fundus images. And this information can better depict vessel details. Contrarily, this information may be lost at the bottom layers (i.e., TransL3). This phenomenon is more evident in the Se and AUC metrics. Similar results can be observed on STARE. Second, we need not add too many Transformer modules into the skip connection. The worst performance is observed when we use three Transformer modules, especially for DRIVE and STARE. On the other hand, too many Transformer modules also need extra computing resources. Certainly, the combination of TransL2 and TransL4 is a good choice if we intend to use many more Transformer modules. This indicates that we should consider both top and bottom information to better complete vessel segmentation. It is a valuable conclusion that is closer to people's objective cognition.

In summary, we should tune the number and position of the plug-and-play Transformer module carefully to obtain the best segmentation performance.

#### 4.4.2. Real Contribution of Each Module

TiM-Net consists of several key components, such as the backbone, dual-attention (DA) mechanism, and Transformer module. Each component acts its role in retinal vessel segmentation. In this subsection, we evaluate the real contribution of each component. And we get a group of model variants by ablation analysis. This helps us recognize the bottleneck of TiM-Net and light our future research. We use Acc, Se, Sp, and AUC metrics to evaluate each model variant. All the results are shown in Table 7. We call this procedure coarse-grained ablation analysis. Here, “Backbone1” represents U-Net [7]. “Backbone2” represents M-Net [17]. “DA” represents the dual-attention mechanism. “TransL2” is the Transformer module. Meanwhile, fine-grained ablation analysis results are shown in Figures 9 and 10.  Figure 9 illustrates the average performance improvement of each model variant on each metric relative to “Backbone1.” Figure 10 illustrates the corresponding performance improvement relative to the “Backbone2.” For example, the average improvement of “DA” on the Se metric relative to “Backbone1” is calculated as follows: ((0.7787 − 0.7042) + (0.7303 − 0.7430) + (0.8132 − 0.7371))/3 = 0.0498. Other values are computed in the same way.

As shown in Table 7, for DRIVE, using different backbones leads to different segmentation performances. Compared with “Backbone1,” the corresponding Acc, Se, Sp, and AUC of “Backbone2” improve about 0.36%, 4.72%, −0.08%, and 4.89%, respectively. Similar results can be found on the other two data sets, especially for STARE. These results validate that M-Net is a better and more robust backbone for retinal vessel segmentation.

Second, for the challenging DRIVE data set, using the dual-attention mechanism leads to evident improvements. Compared with “Backbone1,” the corresponding Acc, Se, Sp, and AUC of “Backbone1 + DA” improve about 0.34%, 7.45%, −0.37%, and 2.28%, respectively. Compared with “Backbone2,” the corresponding Acc, Se, Sp, and AUC of “Backbone2 + DA” improve about 0.29%, 3.55%, −0.36%, and 0.15%, respectively. Similar results can be observed on the other two data sets, especially for STAR. For STARE, compared with “Backbone2,” the corresponding Acc, Se, Sp, and AUC of “Backbone2 + DA” improve about 0.21%, 1.83%, 0.07%, and 0.47%, respectively. Hence, similar to M-Net, the dual-attention mechanism also plays an important role in TiM-Net.

Third, applying the Transformer module leads to evident performance improvements. For STARE, compared with “Backbone2,” the corresponding Acc, Se, Sp, and AUC of “Backbone2 + TransL2” improve about 0.14%, 0.94%, 0.05%, and 0.67%, respectively. Similar results can be observed in the other two data sets. However, compared to the “Backbone2” and dual-attention mechanism, the Transformer module plays a relatively secondary role in our model. Hence, the “Backbone2” and dual-attention modules are more important for retinal vessel segmentation. This also informs us to modify the pure Transformer structure in our future work. All the above discussions belong to the scope of coarse-grained ablation analysis.

Besides coarse-grained ablation analysis, we also make fine-grained ablation analyses to better understand the real contribution of each module. As shown in Figure 9, in terms of AUC, using the “DA” or “TransL2” module can attain more evident performance improvement in Backbone1. Each module improves a specific evaluation metric. In terms of Acc, adding both the “DA” and “TransL2” modules leads to more evident performance improvement. Summarily, each module contributes to promoting the final performance in the Backbone1.

As shown in Figure 10, in terms of Se, using the “DA” module causes the largest performance improvement in Backbone2. This indicates that the “DA” module improves the FNR of the proposed segmentation model. More vessels are segmented accurately by TiM-Net. This may offer more detailed vessel information for the clinical diagnosis. According to Sp, using the Transformer module obtains the best performance. More background pixels are segmented accurately by TiM-Net. We infer this is mostly due to the long-range relationship captured by the MSA mechanism. The combination of the DA and Transformer modules achieves the best AUC improvement. Notably, compared with Figure 9, more balanced improvements are observed by using the “DA” and “TransL2” modules. Hence, we combine the two modules arbitrarily to obtain the best performance. The Transformer and “DA” modules are plug-and-play, which firmly supports this requirement.

Summarily, according to the fine-grained ablation analysis, second only to Backbone2, “DA” plays a more significant role in TiM-Net. Certainly, the combination of the “DA,” “TransL2” modules gets the best overall performance in Backbone2. This can firmly support clinical diagnosis. Moreover, these results are consistent with those of coarse-grained ablation analysis.

## 5. Conclusion and Future Work

We propose a novel model, called TiM-Net, for effective retinal vessel segmentation. To fully use multiscale information, TiM-Net employs the multiscale images after maximum pooling as its inputs. Then the dual-attention mechanism is placed behind the encoder to lower the negative influence of noisy features. Meanwhile, we make feature re-coding using the MSA mechanism of the Transformer module to capture the long-range relationship in the fundus images. Finally, we create a weighted SideOut layer to complete the final segmentation.

We evaluate TiM-Net on the DRIVE, STARE, and CHASEDB1 data sets. They cover diverse diseases, data distributions, and image sizes, which have certain clinical and technological values. Compared with state-of-the-arts, TiM-Net, including its variants, achieves competitive segmentation performance. We make detailed ablation analyses from coarse- and fine-grained perspectives. The descending order of the real contribution of all the modules is “Backbone2 > DA > TransL2.” Notably, we can obtain satisfactory results without any data preprocessing steps, which have certain practicality for clinical diagnosis. Last but not least, in terms of qualitative results, our model has an evident advantage in the segmentation of the disease images, which will be beneficial for the clinical diagnosis. Summarily, owing to satisfactory performance, TiM-Net provides firm technical support for clinical human-computer interaction diagnosis. And it shows clinically satisfactory accuracy and sensitivity to some degree.

Certainly, current researches including the proposed TiM-Net have the following shortcomings: (1) it is difficult to obtain the best performance on each metric; (2) they inevitably lose some vessel details owing to continuous upsampling. Hence, in the future, we plan to modify the internal structure of the Transformer module to improve the corresponding FPR. We intend to get a trade-off between all metrics. Additionally, we will combine the symmetric pattern in Swin-Unet [48] with the coding pattern in MAE [57], to retain sufficient vessel details and make the performance of our model more outstanding on each metric.

## Figures and Tables

**Figure 1:** Structure of TiM-Net. Each layer is marked with the corresponding feature map size and the number of channels. The green block on the left side represents the continuous encoding, and the green block on the right side represents the continuous decoding.

**Figure 2:** Overview of the Transformer: (a) the module structure of the Transformer and (b) the internal structure of each Transformer layer.

**Figure 3:** The proposed dual-attention module. Feature maps pass through serial channel attention and spatial attention one by one after convolution. ⊗ represents the multiplication operation of the corresponding elements, and ⊕ denotes the addition operation of the corresponding elements.

**Figure 4:** The channel attention module.

**Figure 5:** The spatial attention module.

**Figure 6:** Qualitative comparisons with baseline approaches. Our method obtains fewer FPR and retains finer vessel details.

**Figure 7:** Qualitative comparisons between disease and nondisease cases on DRIVE.

**Figure 8:** The average performance improvement of each metric in all the data sets.

**Figure 9:** The average performance improvement of each metric using the Backbone1 (U-Net) in all the data sets.

**Figure 10:** The average performance improvement of each metric using the Backbone2 (M-Net) in all the data sets.

**Table 1:** Performance comparisons on STARE. The best result of each metric is shown as **0.9711**. “—” means that the corresponding value was not provided.

Model	Acc ↑	Se ↑	Sp ↑	AUC ↑
U-Net [7] (2015)	0.9674	0.7371	0.9878	0.8855
Orlando's model [52] (2017)	—	0.7680	0.9738	—
Yan's model [53] (2018)	0.9612	0.7581	0.9846	0.9801
Yan's model [54] (2018)	0.9638	0.7735	0.9857	0.9833
M-Net [17] (2018)	0.9701	0.7446	0.9908	0.8848
DUNet [9] (2019)	0.9641	0.7595	0.9878	0.9832
IterNet [22] (2020)	0.9701	0.7715	0.9886	**0.9881**
EfficientNet [55] (2020)	0.9569	0.7554	**0.9970**	—
TiM-Net-1	0.9674	**0.8109**	0.9819	0.9454
TiM-Net-2	**0.9711**	0.7867	0.9880	0.9670

**Table 2:** Performance comparisons on CHASEDB1. The best result of each metric is shown as **0.9711**.

Model	Acc ↑	Se ↑	Sp ↑	AUC ↑
U-Net [7] (2015)	0.9684	0.7430	0.9842	0.8902
Wu's model [56] (2018)	0.9637	0.7538	0.9847	0.9825
M-Net [17] (2018)	0.9709	0.7606	0.9855	0.8917
DUNet [9] (2019)	0.9610	0.8155	0.9752	0.9804
Wang's model [42] (2019)	0.9661	0.8074	0.9821	0.9812
HANet [21] (2020)	0.9670	0.8239	0.9813	**0.9871**
IterNet [22] (2020)	0.9655	0.7970	0.9823	0.9851
EfficientNet [55] (2020)	0.9643	**0.8477**	0.9825	0.9448
Pyramid U-Net [23] (2021)	0.9639	0.8035	0.9787	0.9832
TiM-Net-1	0.9695	0.7933	0.9814	0.9384
TiM-Net-2	**0.9711**	0.7697	**0.9865**	0.9648

**Table 3:** Performance comparisons on DRIVE. The best result of each metric is shown as **0.9638**.

Model	Acc ↑	Se ↑	Sp ↑	AUC ↑
U-Net [7] (2015)	0.9604	0.7042	**0.9854**	0.9130
Wu's model [56] (2018)	0.9567	0.7844	0.9807	0.9819
M-Net [17] (2018)	0.9634	0.7559	0.9835	0.8985
DUNet [9] (2019)	0.9566	0.7963	0.9800	0.9802
Ma's model [41] (2019)	0.9570	0.7916	0.9811	0.9810
Wang's model [42] (2019)	0.9567	0.7940	0.9816	0.9772
IterNet [22] (2020)	0.9573	0.7735	0.9838	0.9816
HANet [21] (2020)	0.9581	0.7991	0.9813	**0.9823**
TiM-Net-1	0.9616	**0.8033**	0.9770	0.9510
TiM-Net-2	**0.9638**	0.7805	0.9816	0.9682

**Table 4:** The experimental results of assigning the same weight to each layer. The best value of each metric on each data set is shown as **0.9608**.

Data set	Side layer	Acc ↑	Se ↑	Sp ↑	AUC ↑
DRIVE	Side5	0.9233	0.4562	0.9682	0.9026
	Side6	0.9471	0.7107	0.9702	0.9437
	Side7	0.9597	**0.7263**	0.9826	0.9106
	Side8	**0.9608**	0.6944	**0.9868**	0.8944
	SideOut	0.9596	0.7060	0.9844	**0.9529**

STARE	Side5	0.9117	0.6406	0.9355	0.8963
	Side6	0.9421	0.7790	0.9567	0.9451
	Side7	0.9610	**0.7926**	0.9761	0.9191
	Side8	**0.9668**	0.7452	**0.9865**	0.8966
	SideOut	0.9604	0.7783	0.9767	**0.9476**

CHASEDB1	Side5	0.9369	0.6162	0.9582	0.9239
	Side6	0.9569	0.7523	0.9704	0.9491
	Side7	0.9675	**0.7827**	0.9798	0.9295
	Side8	**0.9702**	0.7222	**0.9868**	0.8721
	SideOut	0.9676	0.7527	0.9818	**0.9580**

**Table 5:** The corresponding results of using different weights. The best value of each metric on each data set is shown as **0.9638**. And the improved metric of SideOut compared with Table 4 is shown as **0.9638.**

Data set	Side layer	Acc ↑	Se ↑	Sp ↑	AUC ↑
DRIVE	Side5	0.9278	0.5225	0.9666	0.9195
	Side6	0.9511	0.7578	0.9698	0.9552
	Side7	0.9616	**0.8033**	0.9770	0.9510
	Side8	0.9636	0.7704	**0.9824**	0.8945
	SideOut	**0.9638**	0.7805	0.9816	**0.9682**

STARE	Side5	0.9273	0.5732	0.9594	0.9158
	Side6	0.9522	0.7844	0.9676	0.9549
	Side7	0.9674	**0.8109**	0.9819	0.9454
	Side8	**0.9712**	0.7711	**0.9896**	0.8846
	SideOut	0.9711	0.7867	0.9880	**0.9670**

CHASEDB1	Side5	0.9450	0.5985	0.9683	0.9332
	Side6	0.9617	0.7557	0.9756	0.9519
	Side7	0.9695	**0.7933**	0.9814	0.9384
	Side8	0.**9711**	0.7637	0.9851	0.9141
	SideOut	**0.9711**	0.7697	**0.9865**	**0.9648**

**Table 6:** The ablation analysis results from the application of the Transformer. Our backbone is M-Net [18]. The best value of each metric is shown as **0.9706**.

Data set	TransL2	TransL3	TransL4	Acc ↑	Se ↑	Sp ↑	AUC ↑
DRIVE	✓			**0.9629**	**0.7903**	0.9797	**0.9130**
		✓		0.9627	0.6997	**0.9882**	0.8633
			✓	0.9628	0.7316	0.9852	0.8917
	✓	✓		0.9602	0.7008	0.9857	0.8737
	✓		✓	0.9625	0.7277	0.9853	0.8717
		✓	✓	0.9601	0.6908	0.9862	0.8980
	✓	✓	✓	0.9532	0.6618	0.9813	0.9052

CHASEDB1	✓			**0.9706**	**0.7640**	0.9846	**0.9088**
		✓		0.9702	0.7325	0.9863	0.8847
			✓	0.9705	0.7390	0.9862	0.8806
	✓	✓		0.9686	0.7467	0.9837	0.9113
	✓		✓	0.9696	0.7492	0.8946	0.8738
		✓	✓	0.9678	0.6925	**0.9864**	0.8394
	✓	✓	✓	0.9638	0.6771	0.9832	0.8604

STARE	✓			**0.9700**	**0.7440**	0.9907	0.8705
		✓		0.9685	0.7065	**0.9925**	0.8280
			✓	0.9690	0.7416	0.9899	0.8850
	✓	✓		0.9658	0.7008	0.9901	0.8755
	✓		✓	0.9690	0.7308	0.9908	**0.8937**
		✓	✓	0.9667	0.7028	0.9906	0.8824
	✓	✓	✓	0.9618	0.6465	0.9906	0.8700

**Table 7:** The corresponding coarse-grained ablation analysis results. The best value of each metric is shown as **0.9726**.

Data set	Backbone1	Backbone2	DA	TransL2	Acc ↑	Se ↑	Sp ↑	AUC ↑
DRIVE	✓				0.9604	0.7042	0.9854	0.9130
	✓		✓		0.9638	**0.7787**	0.9817	**0.9358**
	✓			✓	0.9617	0.7136	**0.9858**	0.9345
	✓		✓	✓	**0.9641**	0.7523	0.9847	0.8858
		✓			**0.9640**	0.7514	0.9846	0.9619
		✓	✓		0.9638	**0.7869**	0.9810	0.9634
		✓		✓	0.9639	0.7330	**0.9862**	0.9620
		✓	✓	✓	0.9638	0.7805	0.9816	**0.9682**

CHASEDB1	✓				0.9684	0.7430	0.9842	0.8902
	✓		✓		**0.9713**	0.7303	**0.9874**	0.9172
	✓			✓	0.9693	0.7553	0.9838	**0.9312**
	✓		✓	✓	0.9681	**0.7617**	0.9821	0.9062
		✓			0.9711	0.7523	0.9860	0.9643
		✓	✓		**0.9719**	0.7692	0.9856	**0.9679**
		✓		✓	0.9712	0.7635	0.9854	0.9670
		✓	✓	✓	0.9711	**0.7697**	**0.9865**	0.9648

STARE	✓				0.9674	0.7371	0.9878	0.8855
	✓		✓		**0.9726**	**0.8132**	0.9875	0.9626
	✓			✓	0.9700	0.7681	0.9878	**0.9677**
	✓		✓	✓	0.9697	0.7351	**0.9911**	0.8970
		✓			0.9686	0.7665	0.9871	0.9633
		✓	✓		0.9707	0.7848	0.9878	0.9680
		✓		✓	0.9700	0.7759	0.9876	**0.9700**
		✓	✓	✓	**0.9711**	**0.7867**	**0.9880**	0.9670

## Data Availability

The data that support the findings of this study are openly available at http://cecas.clemson.edu/∼ahoover/stare/, https://blogs.kingston.ac.uk/retinal/chasedb1/, and https://drive.grand-challenge.org/ [48–50].

## References

[1] Reddy G. T., Kaluri R., Reddy P. K., Lakshmanna K., Koppu S., Rajput D. S. (2019). A novel approach for home surveillance system using IoT adaptive security. *SSRN Electronic Journal*.

[2] Kaluri R., Ch P. R. (2018). Optimized feature extraction for precise sign gesture recognition using self-improved genetic algorithm. *International Journal of Engineering and Technology Innovation*.

[3] Zhang H., Liang W., Li C. (2022). DCML: deep contrastive mutual learning for COVID-19 recognition. *Biomedical Signal Processing and Control*.

[4] Fan Z., Lu J., Wei C., Huang H., Cai X., Chen X. (2019). A hierarchical image matting model for blood vessel segmentation in fundus images. *IEEE Transactions on Image Processing*.

[5] Krizhevsky A., Sutskever I., Hinton G. E. (2017). ImageNet classification with deep convolutional neural networks. *Neural Information Processing Systems*.

[6] Long J., Shelhamer E., Long J., Darrell T. Fully convolutional networks for semantic segmentation.

[7] Ronneberger O., Fischer P., Brox T. U-net: convolutional networks for biomedical image segmentation.

[8] Zhou Z., Siddiquee M. M. R., Tajbakhsh N., Liang J. Unet++: a nested U- net architecture for medical image segmentation. *Deep Learning in Medical Image Analysis and Multi-modal Learning for Clinical Decision Support*.

[9] Jin Q., Meng Z., Pham T. D., Chen Q., Wei L., Su R. (2019). DUNet: a deformable network for retinal vessel segmentation. *Knowledge-Based Systems*.

[10] Wang C., Zhao Z., Ren Q., Xu Y., Yu Y. (2019). Dense U-net based on patch-based learning for retinal vessel segmentation. *Entropy*.

[11] Khan T. M., Alhussein M., Aurangzeb K., Arsalan M., Naqvi S. S., Nawaz S. J. (2020). Residual connection-based encoder decoder network (rced-net) for retinal vessel segmentation. *IEEE Access*.

[12] Wu Y., Xia Y., Song Y. Vessel-Net: retinal vessel segmentation under multi-path supervision.

[13] Yu L., Cheng J. Z., Dou Q. Automatic 3D cardiovascular MR segmentation with densely-connected volumetric convnets.

[14] Seo H., Huang C., Bassenne M., Xiao R., Xing L. (2020). Modified U-net (mU-Net) with incorporation of object-dependent high level features for improved liver and liver-tumor segmentation in CT images. *IEEE Transactions on Medical Imaging*.

[15] Xu X., Wang Y., Liang Y. (2022). Retinal vessel automatic segmentation using SegNet. *Computational and Mathematical Methods in Medicine*.

[16] Liu C., Gu P., Xiao Z. (2022). Multiscale U-net with spatial positional attention for retinal vessel segmentation. *Journal of Healthcare Engineering*.

[17] Fu H., Cheng J., Xu Y., Wong D. W. K., Liu J., Cao X. (2018). Joint optic disc and cup segmentation based on multi-label deep network and polar transformation. *IEEE Transactions on Medical Imaging*.

[18] Guo C., Szemenyei M., Yi Y., Wang W., Chen B., Fan C. Spatial attention U-net for retinal vessel segmentation.

[19] Fu J., Liu J., Tian H. Dual attention network for scene segmentation.

[20] Zhang S., Fu H., Yan Y. (2019). Attention guided network for retinal image segmentation. https://arxiv.org/abs/1907.12930.

[21] Wang D., Haytham H., Pottenburgh P., Saeedi S., Tao T. (2020). Hard attention net for automatic retinal vessel segmentation. *IEEE Journal of Biomedical and Health Informatics*.

[22] Li L., Verma M., Nakashima Y., Nagahara H., Kawasaki R. Iternet: retinal image segmentation utilizing structural redundancy in vessel networks.

[23] Zhang J., Zhang Y., Xu X. Pyramid U-net for retinal vessel segmentation.

[24] Chen J., Lu Y., Yu Q. (2021). TransUNet: transformers make strong encoders for medical image segmentation. http://arXiv.org/abs/2102.04306.

[25] Zhang Y., Huiye L., Qiang Hu (2021). TransFuse: fusing transformers and CNNs for medical image segmentation. *MICCAI*.

[26] Chen D., Yang W., Wang L., Tan S., Lin J., Bu W. B. (2022). PCAT-UNet: UNet-like network fused convolution and transformer for retinal vessel segmentation. *PLoS One*.

[27] Zhang J., Jin Y., Xu J., Xu X., Zhang Y. (2018). MDU-Net: multi-scale Densely Connected U-Net for biomedical image segmentation. http://arXiv.org/abs/1812.00352.

[28] Chen W., Zhang Y., He J. Prostate segmentation using 2D bridged U-net.

[29] Devi W. V., Roy S., Thongam K. (2022). Multi-scale dilated fusion network (MSDFN) for automatic instrument segmentation. *Journal of Computer Science and Technology Studies*.

[30] Xu K., Ba J., Kiros R. (2015). Show, attend and tell: neural image caption generation with visual attention. *Computer Science*.

[31] Li C., Tan Y., Chen W. (2020). ANU-Net: attention-based nested U-Net to exploit full resolution features for medical image segmentation. *Computers & Graphics*.

[32] Zhang Z., Lan C., Zeng W., Jin X., Chen Z. Relation-aware global attention for person Re-identification.

[33] Woo S., Park J., Lee J. Y., Kweon I. S. (2018). CBAM: convolutional block Attention module. https://arxiv.org/abs/1807.06521.

[34] Wang F., Jiang M., Qian C. Residual attention network for image classification.

[35] Amer A., Lambrou T., Ye X. (2022). MDA-unet: a multi-scale dilated attention U-net for medical image segmentation. *Applied Sciences*.

[36] Behnke M., Heafield K. Losing heads in the lottery: pruning transformer attention in neural machine translation.

[37] Wang H., Wu Z., Liu Z. (2020). HAT: hardware-aware transformers for efficient natural language processing. http://arXiv.org/abs/2005.14187.

[38] Dosovitskiy A., Beyer L., Kolesnikov A. (2021). An image is worth 16x16 words: transformers for image recognition at scale. https://arxiv.org/abs/2010.11929.

[39] Ye L., Rochan M., Liu Z., Wang Y. Cross-modal self-attention network for referring image segmentation.

[40] Yang F., Yang H., Fu J., Lu H., Guo B. Learning texture transformer network for image super-resolution.

[41] Liu Z., Lin Y., Cao Y. (2021). Swin transformer: hierarchical vision transformer using shifted windows. https://arxiv.org/abs/2103.14030.

[42] Wang B., Qiu S., He H. Dual encoding U-net for retinal vessel segmentation.

[43] Ma W., Yu S., Ma K., Wang J., Ding X., Zheng Y. Multi-task neural networks with spatial activation for retinal vessel segmentation and artery/vein classification.

[44] Tong H., Fang Z., Wei Z., Cai Q., Gao Y. (2021). SAT-Net: a side attention network for retinal image segmentation. *Applied Intelligence*.

[45] Jiang Y., Liu W., Wu C., Yao H. (2021). Multi-scale and multi-branch convolutional neural network for retinal image segmentation. *Symmetry*.

[46] Zhai Z., Feng S., Yao L., Li P. (2022). Retinal vessel image segmentation algorithm based on encoder-decoder structure. *Multimedia Tools and Applications*.

[47] Zhang S., Fu H., Xu Y., Liu Y., Tan M. (2020). Retinal image segmentation with a structure-texture demixing network. https://arxiv.org/abs/2008.00817.

[48] Cao H., Wang Y., Chen J., Jiang D., Zhang X., Tian Q. (2021). Swin-unet: unet-like pure transformer for medical image segmentation. http://arXiv.org/abs/210505537.

[49] Hoover A. D., Kouznetsova V., Goldbaum M. (2000). Locating blood vessels in retinal images by piecewise threshold probing of a matched filter response. *IEEE Transactions on Medical Imaging*.

[50] Owen C. G., Rudnicka A. R., Mullen R. (2009). Measuring retinal vessel tortuosity in 10-year-old children: validation of the computer-assisted image analysis of the retina (CAIAR) program. *Investigative Opthalmology & Visual Science*.

[51] Staal J., Abramoff M. D., Niemeijer M., Viergever M. A., van Ginneken B. (2004). Ridge-based vessel segmentation in color images of the retina. *IEEE Transactions on Medical Imaging*.

[52] Orlando J. I., Prokofyeva E., Blaschko M. B. (2017). A discriminatively trained fully connected conditional random field model for blood vessel segmentation in fundus images. *IEEE Transactions on Biomedical Engineering*.

[53] Yan Z., Yang X., Cheng K. T. (2018). Joint segment-level and pixel-wise losses for deep learning based retinal vessel segmentation. *IEEE Transactions on Biomedical Engineering*.

[54] Yan Z., Yang X., Cheng K. T. (2019). A three-stage deep learning model for accurate retinal vessel segmentation. *IEEE Journal of Biomedical and Health Informatics*.

[55] Mathews M. R., Anzar S. M., Krishnan R. K. EfficientNet for retinal blood vessel segmentation.

[56] Wu Y., Xia Y., Song Y., Zhang Y., Cai W. Multiscale network followed network model for retinal vessel segmentation.

[57] He K., Chen X., Xie S., Li Y., Dollár P., Girshick R. (2021). Masked autoencoders are scalable vision learners. http://arXiv.org/abs/2111.06377.

